The article "Assessing the Nutritional-Value-Based Therapeutic Potentials and Non-Destructive Approaches for Mulberry Fruit Assessment: An Overview" was retracted in 2023. Reasons: unreliable results or conclusions; concerns about the data; concerns about the peer review; concerns about the citations.

# Assessing the Nutritional-Value-Based Therapeutic Potentials and Non-Destructive Approaches for Mulberry Fruit Assessment: An Overview

**DOI:** 10.1155/2022/6531483

**Published:** 2022-03-24

**Authors:** Muhammad Faisal Manzoor, Abid Hussain, Diana Tazeddinova, Aizhan Abylgazinova, Bin Xu

**Affiliations:** ^1^School of Food and Biological Engineering, Jiangsu University, Zhenjiang, Jiangsu, China; ^2^Department of Agriculture and Food Technology, Karakoram International University, Gilgit, Pakistan; ^3^Department of Technology and Catering Organization, South Ural State University, Chelyabinsk, Russia; ^4^Higher School of Technologies of Food and Processing Productions, Zhangir Khan West Kazakhstan Agrarian Technical University, Uralsk, Kazakhstan; ^5^Scientific-Production Center of Livestock and Veterinary Medicine, Nur-Sultan, Kazakhstan

## Abstract

Among different fruits, mulberry is the most highlighted natural gift in its superior nutritional and bioactive composition, indispensable for continuing a healthy life. It also acts as a hepatoprotective immunostimulator and improves vision, anti-microbial, anti-cancer agent, anti-stress activity, atherosclerosis, neuroprotective functions, and anti-obesity action. The mulberry fruits also help reduce neurological disorders and mental illness. The main reason for that is the therapeutic potentials present in the nutritional components of the mulberry fruit. The available methods for assessing mulberry fruits are mainly chromatographic based, which are destructive and possess many limitations. However, recently some non-invasive techniques, including chlorophyll fluorescence, image processing, and hyperspectral imaging, were employed to detect various mulberry fruit attributes. The present review attempts to collect and explore available information regarding the nutritional and medicinal importance of mulberry fruit. Besides, non-destructive methods established for the fruit are also elaborated. This work helps encourage many more research works to dug out more hidden information about the essential nutrition of mulberry that can be helpful to resolve many mental-illness-related issues.

## 1. Introduction

Fruits and vegetables carry health-promoting and bioactive constituents; consequently, consumers' preference has been shifted towards their extensive consumption [1]. Chemical compositions of such food items can protect from various diseases without harming the human body. Mulberry is also a nutritious fruit cultivated 5,000 years ago in China, along with sericulture. Different health-promoting compounds such as moranoline, albafuran, albanol, morusin, kuwanol, calystegine, and hydroxymoricin that can regulate metabolic activities efficiently have been reported [2, 3]. Explorative studies on mulberry fruit have investigated different health-promoting compounds such as moranoline, albafuran, albanol, morusin, kuwanol, calystegine, and hydroxymoricin that can regulate metabolic activities efficiently [4, 5]. In recent years, some reviews were published based on the health benefits of mulberry fruits [6, 7], and only a few studies discussed analysis methods for the mulberry fruit [8]. Moreover, with the recent global increase in demand for nutrient-dense and high-quality foods, there is a strong emphasis on the non-destructive methods of assessment with accuracy and high sensitivity for different phytochemicals. Recently, many reviews have discussed the use of non-destructive spectral imaging and spectroscopic techniques for different food and agricultural applications such as exploring the lycopene content, ripening, and maturity of the fruits and quality assessment of alcoholic beverages and spices [9–11].

The article "Assessing the Nutritional-Value-Based Therapeutic Potentials and Non-Destructive Approaches for Mulberry Fruit Assessment: An Overview" was retracted in 2023. Reasons: unreliable results or conclusions; concerns about the data; concerns about the peer review; concerns about the citations.

Therefore, in the current attempt, we discussed non-destructive and rapid methods for the non-invasive investigation of mulberry samples and also elaborated on the importance of mulberry fruit as a nutritional and health-promoting source.

## 2. Nutritional Significance of Mulberry Fruits

The occurrence of ascorbic acid, carbohydrates, proteins, fats, minerals, and vitamins (thiamine, nicotinic acid, and riboflavin) and their precursors make mulberry fruit the most nutritious agricultural product for consumers [12]. However, a broad range of topographical, climatic, and soil conditions can affect plants' nutritional and chemical status. For example, moisture can range from 80.8 ± 2.81 g/100g FW, ash can vary from 0.6 ± 0.09 g/100g DW, protein can vary from 1.46 ± 0.18 g/100g DW, and the lipid can range from 0.58 ± 0.06 g/100g DW. Likewise, crude fiber (1.2 ± 0.40 g/100 g DW), carbohydrate (15.30 ± 1.27 g/100 g DW), and energy (72.30 ± 3.25 kcal/100 g DW) can also fluctuate [13, 14]. The main sugars are fructose (1.7–2.11 g/100 FW) and glucose (1.7–2.44 g/100 FW) in mulberry fruit. The pH and the total soluble solids (TSS) in mulberry fruit range from 3.23 to 3.42 and 6.19to 9.32, respectively [13, 14].

Moreover, the fruit also contains essential minerals elements (both macro and micro), which aids in regulating metabolic mechanisms. Potassium (K), calcium (Ca), magnesium (Mg), and sodium (Na) are essential elements, while the iron (Fe), zinc (Zn), and nickel (Ni) are among the microminerals reported in different studies [14, 15]. Evaluation of essential minerals in different mulberry varieties from different zones confirmed K as the predominant element, ranging from 906.75 ± 41.49%. Trace elements assessed were ranging in a reasonable amount in the fresh matter, but selenium (Se), arsenic (As), and chromium (Cr) are the least dominant elements [16].

The article "Assessing the Nutritional-Value-Based Therapeutic Potentials and Non-Destructive Approaches for Mulberry Fruit Assessment: An Overview" was retracted in 2023. Reasons: unreliable results or conclusions; concerns about the data; concerns about the peer review; concerns about the citations.

In mulberry fruit, 18 different amino acids were also determined, among which 9 were the essential amino acid compulsory for our body. According to the protein ratio, mulberry fruit is close to the sound quality protein foods such as milk and fish. In mulberry essential, amino acid/total amino acid (EAA/TAA) ratio is about 42% [17]. Similarly, in mulberry fruit, the polyunsaturated fatty acid (PUFA) content is higher than monounsaturated and saturated fatty acids. Moreover, behenic acid (C22: 0) and palmitoleic acid (C16: 1) are essential fatty acids reported in mulberry fruits only. All the reported fatty acids in the fruit are displayed in Table 1.

Additionally, the mulberry fruit also contains riboflavin, thiamin, folate, niacin, and vitamins B-6, A, K, and E. Ascorbic acid is higher, ranging from 36 to 36.4 mg/100/g [20]. Similarly, tocopherols were also revealed by Gómez-Mejía et al. [23] in mulberry fruit, including *α*-tocopherol (0.73 mg/100 g FW), *δ*-tocopherol (2.2 mg/100 g FW), and *γ*-Tocopherol (25 mg/100 g FW). Besides, the fruit also carries organic acids [22], making it a valuable, healthy product, and plays a vital role in sensory properties by imparting sugar and sour taste. Acids are primarily used as an additive, specifically acidulates (malic, tartaric, ascorbic, and citric acids), anti-oxidants (malic, tartaric, and citric acids), or preservatives (benzoic and sorbic acids) [24]. Fruits' base acids have no adverse health effects because during the metabolism they are quickly oxidized. Other vitamins and organic acids present in the fruit are presented in Table 1.

## 3. Phytochemicals in Mulberry Fruit

Non-nutritive phenolic compounds protect from various dysfunctions with no side effects to the consumer's health [25]. The polyphenolic content reported in mulberry fruit includes flavonoids, fibers, *β*-carotene, anthocyanins, anthraquinone, glycosides, and oleic acid [2, 7] (Figure 1). Berries are a good source of polyphenolic and indicate the large family, categorized by the structural attribute as phenolic acids, flavonoids, tannins, stilbenes, and lignans, which are indispensable for life [7]. In mulberry fruits, the phenolic contents fluctuate with various cultivars. Beyond the cultivars, the maturity stages of mulberry fruits also have a notable influence on the phenolic values. With the increase in the maturity stage of mulberry fruit, phenolic content also enhances [12, 26].

### 3.1. Flavonoids

Flavonoids are among a large group of non-nutritive polyphenolic compounds that exhibits anti-oxidant attributes that play a pivotal role in curing oxidative stress-related problems such as atherosclerosis [27]. The variation in flavonoids contents in various breeds of mulberries is notable. Chinese mulberries have higher flavonoid contents (0.0024 mg/kg) than Korean (0.0006 mg/kg) [18]. Quercetin 3-O-*β*-D-(6″-O-malonyl) glucoside is the most important flavonoid for delivering anti-oxidant properties in the fruit [28]. The kaempferol 3-O-glucoside content was observed in mulberry to be 3.55–47.80 mg/kg of fresh weight in *Morus atropurpurea* cv Taiwanguosuang and Yuefenshen [29]. Besides, mrin (flavonoid) was also revealed to suppress cyclosporine in tissues. Cyclosporine is an effective immune suppressive agent that reduces nitric oxide creation by the activated macrophages [30]. Studies also demonstrated inhibition of the human cytochrome CYP3A process in a pooled human liver microsome system by regular consumption of black mulberry fruit juice [31]. Studies conducted on mice also confirmed anti-stress activity in black mulberry juice due to its valuable phytochemical composition [32].

The article "Assessing the Nutritional-Value-Based Therapeutic Potentials and Non-Destructive Approaches for Mulberry Fruit Assessment: An Overview" was retracted in 2023. Reasons: unreliable results or conclusions; concerns about the data; concerns about the peer review; concerns about the citations.

### 3.2. Anthocyanins

Anthocyanins are color imparting pigments, widely distributed in agricultural products including fruits, vegetables, flowers, and others [33]. Numerous studies confirmed the presence of health-promoting anthocyanins in mulberry fruit juice. Among them, cyanidin-3-O-glucoside and cyanidin-3-rutinoside are widely distributed (Table 2) [41].

Moreover, cyanidin 3-O-*β*-D-glucopyranoside isolated from mulberry fruits inhibited the cerebral ischemic damage caused by oxygen-glucose deprivation in PC12 cells [42]. Similarly, anthocyanins from the mulberry fruit (black) were also reported to prevent Cu-induced peroxidation of liposomes [42]. Meanwhile, the co-oxidation of linoleic acid and *β*-carotene confirmed that the extracts of mulberry (*Morus nigra*) fruits show safeguard action against peroxidative damage to biomolecules and their membranes [43]. Furthermore, Jiang et al. [44] and Wu et al. [45] concluded that the fruit anthocyanin and water extract could scavenge free radicals, prevent low-density lipoprotein oxidation, reduce blood lipid, and also be found to prevent atherosclerosis.

### 3.3. Flavonols and Flavanols

Flavonols and flavanols are flavonoids subgroups, and the structures of these flavonoids are almost the same but different in some positions, such as C-2, C-3, and C-4. In flavonols, a double bond exists between C-2 and C-3 and, in the C ring, the carbonyl group at C-4 compared with flavanols. Mulberry fruit consists of many flavonols such as quercetin, rutin, kaempferol, and myricetin, and the derivatives of kaempferol and quercetin are the main components. Some kaempferol in glycosylated form has been found in some cultivars of mulberry fruit, such as kaempferol 3-O-rutinoside and kaempferol 3-O-glucoside [46, 47]. Usually, the flavanols do not exist as a glycoside naturally. But, in mulberry fruit, epigallocatechin gallate, catechin, procyanidin B1, epicatechin, and procyanidin B2 have been reported (Table 2).

The article "Assessing the Nutritional-Value-Based Therapeutic Potentials and Non-Destructive Approaches for Mulberry Fruit Assessment: An Overview" was retracted in 2023. Reasons: unreliable results or conclusions; concerns about the data; concerns about the peer review; concerns about the citations.

### 3.4. Phenolic Acids

Mulberry fruit consists of different types of phenolic acids. Benzoic acid and hydroxycinnamic acids are the leading derivatives that represent the phenolic acids in the fruit. Ferulic acid, cinnamic acid, chlorogenic acid, o-coumaric acid, caffeic acid, and p-coumaric acid are the leading derivatives of hydroxycinnamic acid found in the samples. The gallic acid, protocatechuic acid, hydroxybenzoic acid, and vanillic acid are the essential derivatives of benzoic acid in mulberry fruit (Table 3). In mulberry fruit, the most abundant phenolic acid is chlorogenic acid ranging from 5.3 to 17.3 mg/100 g DW [49]. Furthermore, Butkhup et al. [40] reported that cinnamic acid varied from 11.63 to 15.04 mg/100 g DW and gallic acid fluctuated from 7.34 to 23.35 mg/100 g DW, which is the most prominent phenolic acids in different cultivars of the fruit.

### 3.5. Polysaccharides

Polysaccharides play significant parts in pathological and physiological activities [50–52]. Different polysaccharides were purified from the mulberry fruit with hypoglycemic and anti-oxidant activities using numerous purification methods as presented in Table 4. A glycoprotein extracted from the lyophilized powder and fruit juice of mulberry fruit exhibit good anti-inflammatory and anti-apoptosis agents in rats' primary splenocytes [54].

## 4. Biosynthesis of Anthocyanin and Phenolic Contents in Mulberry

Anthocyanins are the phenylpropanoid metabolic pathway responsible for exhibiting red, purple, and bluish colors to the mulberry fruits. Its biosynthesis begins with amino acid phenylalanine that is converted by phenylalanine ammonia-lyase (PAL), cinnamate 4-hydroxylase (C4H), and 4-coumarate-CoA ligase (4CL) to *ρ*-coumaroyl-CoA (anthocyanin, flavonols, and lignins precursor). Anthocyanins (cyanidin 3-O-rutinoside) are primarily synthesized by chalcone synthase (CHS), chalcone isomerase (CHI), flavanone-3-hydroxylase (F3H), flavonoid-3′-hydroxylase (F3′H), dihydroflavonol reductase (DFR), anthocyanidin synthase (ANS), anthocyanidin 3-O-glucosyltransferase (3GT), and UDP-rhamnose: anthocyanidin-3-glucoside rhamnosyltransferase (3RT). This biosynthesis is regulated by transcription factors (TFs), including MYB and basic helix-loop-helix (bHLH) TFs and WD40-repeat proteins also [59]. Cyanidin-3-rutinoside and cyanidin-3-glucoside are the major anthocyanins isolated from mulberry fruits [59].

The article "Assessing the Nutritional-Value-Based Therapeutic Potentials and Non-Destructive Approaches for Mulberry Fruit Assessment: An Overview" was retracted in 2023. Reasons: unreliable results or conclusions; concerns about the data; concerns about the peer review; concerns about the citations.

Among flavonoids, rutin, quercetin, and kaempferol are the major existing ones in mulberry fruits. Some mulberry cultivars have been reported with glycosylated forms of quercetin and kaempferol, including quercetin 3-O-rutinoside, quercetin 3-O-glucoside, quercetin 3-O-galactoside, kaempferol 3-O- glucoside, and kaempferol 3-O-rutinoside [20]. Moreover, rutin was reportedly the most abundant phenolic acid contributing approximately 44.66% of the total phenolic acid content in eleven different mulberry fruit samples [20].

## 5. Mulberry Homeostasis in Human Guts

The gut response was observed in evaluating anti-oxidant studies (ABTS and FRAP) of mulberry cultivars, whereas, on stimulation of gastrointestinal digestion, white mulberry cultivars exhibited insufficient anti-oxidant activity as compared to their black counterparts. Compared with FRAP assay, white cultivars on digestion possess better anti-oxidant capacity, while the black cultivar showed better results in the non-digested form [60]. Human gut microbiota fermentation effect on the anti-oxidant and phenolic content was observed, where the black mulberry variety showed higher anti-oxidant activity than white in ABTS scavenging activity, while, for the FRAP assay, ferric reducing capacity showed fluctuations in results collected at 0, 2, 6, 12, and 48 hours. Similarly, the phenolic acid content decreased after fermentation in white while in black initially increased to 960.42 mg gallic acid equivalent (GAE)/100 g FW 24 hours. Still, it then significantly decreased to 543.03 GAE at 48 hours. Anthocyanins were also reportedly increased at 0 h, but with a change in pH, a structural modification was observed during fermentation producing different phenolic metabolites. After in vitro digestion, mulberry anthocyanins degraded owing to the alkaline condition of intestinal digestion. Studies showed that acidic pH was considered more stable for anthocyanins' structural integrity [60, 61]. Studies indicate the potential of digested and fermented mulberry samples in suppressing the outbreak of reactive oxygen species (ROS), as highlighted in Figure 2 [62]. Anthocyanins and catechins also act as a cellular signaling messenger to regulate the anti-oxidant enzymes and activate the Keap1/Nrf2 signaling pathway that could increase the gene expression of anti-oxidant enzymes and resultantly maintain the cellular redox balance [60, 63]. Black mulberry cultivars exhibited higher bioactive compounds with potent in vitro anti-oxidant activity and cellular ROS scavenging activity among the different tested cultivars.

The article "Assessing the Nutritional-Value-Based Therapeutic Potentials and Non-Destructive Approaches for Mulberry Fruit Assessment: An Overview" was retracted in 2023. Reasons: unreliable results or conclusions; concerns about the data; concerns about the peer review; concerns about the citations.

## 6. Medicinal Value

Due to the health-promoting nutritional composition of mulberry fruit, its applications extend to medicine, economic enhancement, industrial by-products, clinical and domestic fields [32, 42]. Numerous authors stated that mulberry (fruit, roots, and bark) has vital importance in Chinese folk medicine, reported using since 659 AD for the treatment of different ailments such as preventing diabetes, anemia, hypotension, anti-phlogistic, hepatoprotective, diuretic, hypotensive, anti-pyretic, analgesic, expectorant, and also effective against arthritis [18, 64–67]. Furthermore, the fruit and its extracts are useful against epileptic convulsions, mental problems, and hemicranias. The fruit can also prevent asthma, vitiated conditions, rheumatism, and inflammatory issues [42].

Nonetheless, for many years, mulberry fruit juice has also been consumed as a folk medicine for tumors of fauces, diarrhea, aphtha, flue, cough, dyspepsia, edema, fever, headache, hypertension, and rapid healing of injuries [68]. Moreover, mulberry juice is provided in febrile disorder and malaria to reduce the body temperature because the juice (mulberry) is a natural refrigerant [69]. Similarly, the products (especially syrups and recipes) prepared using mulberry fruits effectively alleviate constipation problems, insomnia, premonitory, and apoplexy dysfunctions [31].

Moreover, the fruit is also effective in treating loss of appetite problems, flatulence, controlling intestinal parasites, and, most importantly, improving the production of body fluids. Different experiments also proved its anti-hyperlipidemic properties, hypertension preventive agent, anti-hyperglycemic, and anti-allergic properties (Table 5) [7, 32, 33, 42, 69].

Chinese pharmacopeia enlists all parts of mulberry (fruit, root bark, stem, and leaves) as a critical constituent in medicinal preparations [84, 85]. Additionally, it poses an anti-aging effect and imparts positive effects on blood lipid and atherosclerosis [86]. This widely grown fruit also has corrective action against bronchitis, edema, influenza, eye infections, and nosebleeds [85]. Traditionally, mulberry can also be used to treat weakness, fatigue, premature hair falling and graying, urinary problems, tinnitus, dizziness, and hypoglycemic action [42]. In contemporary medicine, mulberry is used to prepare oral syrups, add flavor, or impart color to different drugs [87].

### 6.1. Anti-Oxidant Potential

Natural anti-oxidants in produce continuously inactivate the reactive species (which damage cells) and keep them in minor amounts, required for normal cell functioning [88]. The in vitro free radical's assays are the most generally employed methods in estimating the anti-oxidant potential of mulberry fruits (Table 6). Generally, the anti-oxidant activity of the whole frozen fruits was 0.21–8.15%, 50.18–86.79%, 16.53–62.83%, and 0.03–38.45 *μ*M ascorbic acid by using a metal chelating ability, DDPH activity, superoxide anion radical scavenging methods, and FRAP activity, respectively [93]. Different experiments have concluded that fruits containing anti-oxidant compounds significantly reduce specific chronic ailments [94]. Berthollide compounds, one of the secondary metabolites, were also detected in mulberry fruits. These bioactive ingredients are free radical scavengers to protect the cell from oxidation [95]. According to another study, the fruit also strengthens the oxidation safeguarding mechanism and inactivates the red-blood-cell-damaging ingredient in diabetes-induced mice [96].

The article "Assessing the Nutritional-Value-Based Therapeutic Potentials and Non-Destructive Approaches for Mulberry Fruit Assessment: An Overview" was retracted in 2023. Reasons: unreliable results or conclusions; concerns about the data; concerns about the peer review; concerns about the citations.

Moreover, research was conducted to compare the anti-oxidant potential of different fruits. Among the tested samples, the mulberry pulp was characterized highest anti-oxidant (ferric reducing the power of 4.11 mmol/100 g wet weight) exhibiting fruit [97]. Furthermore, a spectroscopic assessment also showed the fruit juice contains efficient scavenging characteristics against superoxide, hydroxyl, and nitric acid.

### 6.2. Immunostimulator

The immune system (IS) is the primary regulatory system managing the body's homeostasis and plays an essential part in developing life from childbirth to death. The IS can be balanced and guarded by using different immunostimulators. Mulberry carries a more significant amount of bioactive flavonoids, particularly anthocyanins and other bioactive compounds that play an essential role in improving the consumer's immunity [98]. *Morus alba* extracts also improved cell-mediated and humoral immunity during experimental animal studies [99].

### 6.3. Anti-Cancer Agent

Cancer disease is one of the main reasons for the death of both humans and animals [100]. Anthocyanins extracted from the mulberry fruit exhibit inhibitory results on migration and invasion of highly metastatic A549 carcinoma cells (human lung) in a dose-dependent method [64]. The methanolic extract of *M. alba* subdued the production of tumor necrosis factor-*α* (TNF-*α*) in macrophages. It inhibited or blocked the production of nitrogen oxide, which was LPS-activated RAW2647 [101]. Mulberry fruit extracted hydroxycinnamic acid derivatives to enhance ROS production by playing as pro-oxidants and destroying the cancer cells [102]. In another study, Huang et al. [79] proposed that mulberry anthocyanins suppressed tumorigenesis and cell survival in AGS gastric cancer xenograft model cells by attacking the c-jun and p38/p53 signaling pathways. Besides, more clinical trials and evaluations verified the curative properties of anthocyanins toward cytotoxic cells, a low-cost and readily accessible source for cancer medication, and decreased cancerous cells [103].

The article "Assessing the Nutritional-Value-Based Therapeutic Potentials and Non-Destructive Approaches for Mulberry Fruit Assessment: An Overview" was retracted in 2023. Reasons: unreliable results or conclusions; concerns about the data; concerns about the peer review; concerns about the citations.

### 6.4. Hepatoprotector

The liver is one of the essential organs in the human body responsible for nutrients, growth, biochemical pathways, energy supply, and several other basic mechanisms. Hepatotoxins are dangerous elements that can harm the liver [104]. Some specific bioactive compounds in mulberry fruit, such as coumarin, flavonoids, anthocyanins, and stilbenes, were described to own hepatoprotective activity [67]. Furthermore, the hydroalcoholic extract of mulberry was verified to decrease isoniazid-produced hepatotoxicity, a specific enzyme (alanine aminotransferase and aspartate aminotransferase) deficiency ailment [105].

### 6.5. Atherosclerosis

Atherosclerosis is the deposition of hard yellow plaques of cholesterol in arteries' inner layers, producing heart attack or coronary thrombosis. Investigations on human health proved that dietary intake of natural anti-oxidants inhibits coronary cardiovascular diseases. Oxidation of low-density lipoprotein (LDL) and cholesterol deposition are two essential factors of atherosclerosis. Though, anti-oxidants supplementation could reduce the growth of atherosclerosis ailments [106]. Valuable bioactive compounds such as quercetin and anthocyanins are proclaimed for their shielding effects as anti-oxidant nutrients. Quercetin and its conjugates are principal representatives of the flavonol group of the mulberry; flavonols have potent inhibitory results on oxidative modification of human LDL in vitro [107]. Liu et al. [108] examined the mulberry anthocyanin extract (MAE) and mulberry water extracts (MWE) for the anti-atherosclerosis effect in vitro. The MAE and MWE scavenged the DPPH radicals and repressed the electrophoretic mobility, the production of thiobarbituric acid reactive substances, and Cu^2+^ induced ApoB fragmentation in oxidation LDL (*p* < 0.05). MAE and MWE also suppress the formation of foam cells and oxidative LDL-induced macrophage death (*p* < 0.05).

### 6.6. Neuroprotective

According to studies, one of the principal causes of neurodegeneration is caused by free radicals [109]. In mulberry fruit, the occurrence of cyanidin and its 3-O-*β*-D-glucopyranoside (Cyn3-O-*β*-D GP) compounds protect consumers against cerebral ischemia [7]. Cyn3-O-*β*-D GP is a prominent neuroprotective component of mulberry fruit extract [82]. Furthermore, Cyn3-O-*β*-D GP has free radical scavenging and inflammation suppressing activity and protects the brain from endothelial dysfunction [110]. Similarly, mulberry fruit extract and Cyn3-O-*β*-D GP can prevent reactive oxygen species production and suppress neuronal disorders. Moreover, in PC12 (oxygen-glucose-deprived) cells, Cyn3-O-*β*-D GP improves the viability of cells and acts as a neuroprotector against cerebral ischemia.

The article "Assessing the Nutritional-Value-Based Therapeutic Potentials and Non-Destructive Approaches for Mulberry Fruit Assessment: An Overview" was retracted in 2023. Reasons: unreliable results or conclusions; concerns about the data; concerns about the peer review; concerns about the citations.

### 6.7. Hypolipidemic and Anti-Obesity Action

The anti-obesity activity of mulberries was conducted both in animal and cell models by various mechanisms (Figure 2). Obesity is defined as an elegant fat collection that increases the risk of health. Obesity hurts diabetes, hypercholesterolemia, atherosclerosis, hepatic steatosis, and hyperlipidemia and reduces the number of sugar absorption that ends in body weight. Research on mulberry extract showed the inverse relationship on the melanin-concentrating hormone (MCH) receptor, which is very helpful to reduce body weight [111]. MWE consists of polyphenols such as chlorogenic acid, gallic acid, anthocyanins, and rutin. MWE reduced visceral fat, body weight induced by a high-fat diet accompanied by hypolipidemic effects by lowering cholesterol, serum triacylglycerol, the LDL/HDL ratio, and free fatty acid. Protect the liver from impairment by lowering the hepatic lipids. In a study, MWE significantly raised the receptor *α* and carnitine palmitoyltransferase-1 of the hepatic peroxisome, while 3-hydroxy-3-methylglutaryl−coenzyme A reductase and fatty acid syntheses enzymes were suppressed. The results indicated that the MWE regulates lipolysis and lipogenesis that eventually imparts hypolipidemic and anti-obese effects [77]. Lately, the mulberry anti-obesity mechanism was revealed. The illustrative mulberry anthocyanin could improve the mitochondrial function via the p38-AMPK-PGC1*α* pathway [112]. Moreover, mulberry pelargonidin and cyanidin controlled various obese signs in male C57BL/6 mice, including a high-fat intake [113]. Peng et al. [77] described that after six weeks of feeding with polyphenol-rich extracts of mulberry, the free fatty acids and bodyweight of high-fat intake old male hamsters were decreased.

## 7. Non-Destructive Techniques and Food Quality Evaluation

With the rapid increase in population and awareness, good quality food is an emerging challenge globally. Therefore, researchers focus on establishing reliable approaches for authenticating agricultural products' quality parameters, including internal and external attributes. Non-destructive powerful spectroscopic techniques have been studied for applications in milk, fish, meat, fruit, vegetable, and beverages [114–118]. The spectral imaging technique is also an accessible option, which combines digital imaging and spectroscopic techniques to provide a powerful analytical device. Such imaging approaches can deliver both spatial and spectral information simultaneously, enabling the detection of the sample down to molecular levels [11, 119].

The article "Assessing the Nutritional-Value-Based Therapeutic Potentials and Non-Destructive Approaches for Mulberry Fruit Assessment: An Overview" was retracted in 2023. Reasons: unreliable results or conclusions; concerns about the data; concerns about the peer review; concerns about the citations.

Non-destructive assessment techniques are the central part of high-quality control functions, and they assist the different established techniques as well. Non-interruptive examination leads to the surface testing of agricultural products without any interfering technique concerning the food quality and appearance. These techniques provide data on food properties such as mechanical, chemical-physical, and structural properties. The employment of a non-destructive assessment is the most suitable way for food processing [120]. Agricultural products possess anti-oxidant attributes due to bioactive compounds such as lycopene, anthocyanins, quercetin, and polyphenols, preventing cellular oxidation. However, these functional components are highly unstable and can be destroyed by conventional methods such as high-performance liquid chromatography, gas chromatography, thin-layer chromatography, and other techniques. Therefore, to ensure the quality assessment of such nutritious compounds, non-destructive spectroscopic and imaging methods are the best available options.

### 7.1. Non-Destructive Technique and Mulberry Fruit Assessment

#### 7.1.1. Chlorophyll Fluorescence (CF)

CF estimation is a non-interruptive and straightforward tool, widely applied to calculate the degree of pigment changes during ripening stages of different agricultural products [121]. In general, the light absorbed by photosynthetic organisms (using chlorophyll) can undergo three different pathways, whether it can be employed to carry out the photosynthesis process result in heat production, or reemitting fluorescence (red). All the operations occur in the competition; therefore, an increase or decrease in one pathway affects the intensity of others. Moreover, estimation of the total yield of fluorescence (chlorophyll) can provide information about changes in the power of photochemistry and heat generation (Figure 3(a)) [124, 125].

Handheld equipment is cost-effective and readily available in the market. Numerous studies have been reported recently using CF to monitor the ripening stages of fruits, including tomato fruit [124], jujube (*Ziziphus jujuba* Mill.) [126], and tobacco seeds [127].

Furthermore, in another study, CF measurements and red, green, and blue (RGB) intensity were used to investigate sugars, total phenols, ABTS cation, total flavonoid, and DPPH radical scavenging properties during different ripening stages non-destructively. The fitted relationship showed a high correlation relationship between CF and RGB intensities with the tested parameters. A high correlation between CF and tested parameters was estimated from 0.82 to 0.94 during the 4–7 ripening stages, while the correlation between RGB and internal tested parameters (*R*^2^) fluctuated from 0.93 to 0.97 for stages 4–7. The study concluded that the CF and RGB intensity values could non-destructively and rapidly assess the quality of fruits during different ripening stages [128].

The article "Assessing the Nutritional-Value-Based Therapeutic Potentials and Non-Destructive Approaches for Mulberry Fruit Assessment: An Overview" was retracted in 2023. Reasons: unreliable results or conclusions; concerns about the data; concerns about the peer review; concerns about the citations.

#### 7.1.2. Image Processing (IP)

In recent years, a combination of machines proved promising in different research areas. For example, machine vision integrated with artificial intelligence delivered the best results for identifying and classification quality attributes of agricultural commodities [123, 129]. Besides, IP and machine vision also aid in the quality control of food items with high accuracy and rapidness and in a non-destructive manner [130, 131]. Numerous research works have been conducted using machine vision efficiently on different fruits and vegetables such as date [132], carrot [133] apples [134], banana [135], potato [136], olive [137], and pomegranate [138]. The main components of a typical IP and essential steps are presented in Figure 3(b).

Similarly, a study was also designed for grading mulberry fruits based on maturity (ripe, unripe, and overripe) using IP and classification methods. Each segmented sample's color and textural attributes were extracted by employing a correlation-based feature selection subset (CFS) and consistency subset (CONS) as two different feature reduction models. Simultaneously, artificial neural networks (ANN) and support vector machines (SVM) were helpful in the sample classification. ANN classification combined with the CFS subset feature extraction method delivered accuracy of 100%, 100%, and 99.1% and the least mean square error (MSE) calculations of 9.2 × 10^−10^, 3.0 × 10^−6^, and 2.9 × 10^−3^ for training, validation, and test sets, respectively. Moreover, the ANN approach integrated with the CONS subset feature extraction approach delivered an acceptable model with the accuracy recorded as 100%, 98.9%, and 98.3%, and MSE resulted as 4.9 × 10^−9^, 3.0 × 10^−3^, and 3.1 × 10^−3^ for training, validation, and test sets, respectively, in a study [138].

#### 7.1.3. Hyperspectral Imaging (HSI)

A combination of spectral and imaging tools proved promising in numerous food applications recently. The method's sensitivity is due to the generation of three-dimensional data cubes by converting spectral information into spatial data. Hence, HSI can provide a spatial map composed of spectral variations at each pixel [139]. The vibrational attributes of C–H, H–O, C–O, and N–H bonds in the food system can be easily studied by employing the HSI system [140]. Compared to traditional computer vision and human vision, the HSI system has natural advantages that can highlight some of the problematic or impossible features to extract with conventional computer vision systems [141, 142]. With the advancement in optical sensing and imaging approaches, the HSI system has recently become a scientific and effective tool for monitoring and evaluating the quality of fruits and vegetables. The main components of a typical HSI are presented in Figure 3(c).

The article "Assessing the Nutritional-Value-Based Therapeutic Potentials and Non-Destructive Approaches for Mulberry Fruit Assessment: An Overview" was retracted in 2023. Reasons: unreliable results or conclusions; concerns about the data; concerns about the peer review; concerns about the citations.

Due to its high sensitivity and non-destructive nature, HSI was employed to detect different constituents in complex food matrices. For example, visible and near-infrared (Vis-NIR) HSI (covering 400–1,700 nm range) has been investigated for non-destructive pectin polysaccharides detection in Dashi and Guihuami intact mulberry varieties. Also, four types of pectins (DASP, WSP, CSP, and TSP) were stored in the room and at low temperatures to analyze the prediction efficiency. Results revealed easier detection of pectins in Dashi samples than others, and the samples stored at room temperature delivered good prediction compared to low temperature stored samples [143]. Similarly, total anthocyanin values and anti-oxidant attribute was also determined by Huang et al. [144] in mulberry fruit using the Vis-NIR HSI method. The best prediction method for total anthocyanins and anti-oxidant property showed *R*^2^_val_ of 0.959 and 0.995, and RPD was calculated as 4.96 and 14.25, respectively. Moreover, the non-destructive method was also used to monitor various pectins in mulberry fruits at different storage temperatures. Dilute alkali-soluble pectin (23.52–91.78 g/kg), water-soluble pectin (17.33–117.44 g/kg), chelator soluble pectin (22.91–135.52 g/kg), and total soluble pectin (63.77–344.75 g/kg) were analyzed in the study. The best prediction outcomes were recorded from dilute alkali-soluble pectin and total soluble pectins in the Dashi cultivar stored at room temperature, delivering satisfactory residual predictive deviation results of 2.31 and 1.93, respectively [145].

## 8. Conclusion and Future Prospects

Investigations on mulberry fruit's health-promoting bioactive compounds proved the disease-fighting attributes in treating various chronic dysfunctions. Clinical trials proved its positive impact against cardiovascular problems, HIV, diabetes, different type of cancers, and obesity and that it can prevent body cell damage, strengthen the nervous system, and can also alleviate many other chronic ailments. Despite these efforts, future work can be focused on the detection of new phytochemicals with more effective and green extraction methods, such as ultrasonication, supercritical fluid extraction, cold plasma method, low polarity water, pulsed electric field, and their integration with other non-thermal methods. In addition, due to the rich phytochemicals and anti-oxidants, the fruit is more worthy for dieticians and health care industries in future research domains. However, some of the polyphenols mechanism in the human body is still not clear yet, need to be thoroughly studied in future works. Furthermore, the stability of polyphenols is also a challenge and further work can be addressed by proposing novel methods in enhancing their stability.

The article "Assessing the Nutritional-Value-Based Therapeutic Potentials and Non-Destructive Approaches for Mulberry Fruit Assessment: An Overview" was retracted in 2023. Reasons: unreliable results or conclusions; concerns about the data; concerns about the peer review; concerns about the citations.

Likewise, fast, green, label-free, and non-destructive methods are also required for accurate and non-interruptive assessment of mulberry fruit attributes. Numerous imaging methods (such as soft X-ray imaging, laser backscattering imaging, multispectral imaging, resonance imaging, thermal imaging, microwave imaging, and others) and spectroscopic approaches such as surface enhance Raman spectroscopy, near-infrared spectroscopy, Fourier transforms infrared spectroscopy, and others may be the smart choice in upcoming projects.

## Figures and Tables

**Figure 1:** Main mulberry functional components and their therapeutic properties.

**Figure 2:** The primary health effects mechanism of mulberry's polyphenols designed from available literature. GSH-Px: glutathione peroxidase, CPT-1: carnitine palmitoyltransferase-1, PGC1*α*: peroxisome proliferator-activated gamma coactivator 1-*α*, PPAR*α*: peroxisome proliferator-activated receptor alpha, UCP1: uncoupling protein 1, PRDM16: PR domain containing 16, HMG-CoA: 3-hydroxy-3-methyl-glutaryl-coenzyme A reductase, SREBP-1c: sterol regulatory element-binding transcription factor 1, LDLR: low-density lipoprotein receptor, AMPK: AMP-activated protein kinase, ABCA1: ATP-binding cassette transporter A1, SR-B1: scavenger receptor class B type 1, GLUT4: glucose transporter type 4, G6Pase: glucose 6-phosphatase, AS160: Akt substrate of 160 kDa, PEPCK: phosphoenolpyruvate carboxykinase, AKT: protein kinase B, FOXO1: fork head box protein O1, GSK-3*β*: glycogen synthase kinase-3*β*, MMPs: matrix metallopeptidases, NF-kB: nuclear factor kappa-light-chain-enhancer of activated B cells, ROS: reactive oxygen species, AP-1: activator protein 1, u-PA: urokinase plasminogen activator, p53: phosphoprotein p53, Apaf1: apoptotic peptidase activating factor 1, Bcl-2: b-cell lymphoma 2, Bace2: beta-secretase 2, AST: aspartate aminotransferase, PI3K: phosphatidylinositol-3 kinase, ALT: alanine aminotransferase, COX 2: cyclooxygenase-2, iNOS: inducible nitric oxide synthases, and ALP: alkaline phosphatase. Note: Orange boxes indicate increase and red boxes indicate decrease.

The article "Assessing the Nutritional-Value-Based Therapeutic Potentials and Non-Destructive Approaches for Mulberry Fruit Assessment: An Overview" was retracted in 2023. Reasons: unreliable results or conclusions; concerns about the data; concerns about the peer review; concerns about the citations.

**Figure 3:** (a)Working mechanism of CF [122], (b)imaging system for mulberry classification [123], and (c)main component of HSI system [1].

**Table 1:** Fatty acid composition, vitamins contents, and organic acids profile in mulberry fruit.

Fatty acid						References
Name		Concentration	Name		Concentration	
Myristic acid		0.47–0.49	Behenic acid		1.3–1.37	[18, 19]
Palmitoleic acid		0.38–0.40	Tetracosanoic acid		1.0–1.04	
Palmitic acid		20–22.26	9-Octadecynoic acid		—	
Heptadecanoic acid		0.26–0.28	10-Nonadecenoic acid		—	
Linoleic acid		26–26.45	Azeloic acid		0.23	
Oleic acid		10.00–10.68	Oxiraneoctanoic acid		0.41	
Stearic acid		8–8.62	11-Eicosenoic acid		—	
Eicosanoic acid		2.10–2.45	Brassidic acid		0.83	
Linolenic acid		0.66	PUFA		74.11–79.52	
MUFA		5.92–6.89	SFA		14.56–19.82	
*Vitamin*						*References*
*Name*	*Concentration*		*Name*	*Concentration*		
Thiamin (B_1_)	0.026–0.029 mg/100 g		Folate DFE^b^	6.00 *μ*g/100 g		[14, 20]
Riboflavin (B_2_)	0.900–0.101 mg/100 g		Vitamin A, RAE^c^	1.00 *μ*g/100 g		
Nicotinic acid	0.700–0.800 mg/100 g		Vitamin A, IU^a^	25 IU/100 g		
Ascorbic acid	36.00–36.40 mg/100 g		Vitamin E (*α*-tocopherol)	0.80–0.87 mg/100 g		
Niacin	0.600–0.620 mg/100 g		Vitamin K	7.60–7.80 *μ*g/100 g		
Vitamin B-6	0.030–0.050 mg/100 g					
*Organic acids*						*References*
*Name*		*Concentration*	*Name*		*Concentration*	
Malic acid		9.095 mg/g	Citric acid		1.805 mg/g	[21, 22]
Tartaric acid		0.145 mg/g	Oxalic acid		0.660 mg/g	
Fumaric acid		0.213 mg/g	Succinic acid		2.836 mg/g	
Lactic acid		0.662 mg/g	Acetic acid		0.053 mg/g	

^*∗*^Fatty acids results: Results are described as percentage over the total peak area content of gas chromatography-mass spectrometry analysis. ^a^IU = international unit, ^b^DFE; dietary folate equivalents, and ^c^RAE; retinol activity equivalents.

**Table 2:** Composition of flavonoids in mulberry fruit.

Class	Subclass	Compound	Contents	References
Flavonoids	Anthocyanins	Cyanidin 3-O-(6″-O-a-rhamnopyranosyl-*β*-D-glucopyranoside)	57 mg/g CMA	[34]
		Cyanidin-3-rutinoside	108.78 mg/g MAE	[35]
		Cyanidin-3-glucoside	301.74 mg/g MAE	[36]
		Cyanidin 3-O-(6″-O-*α*-rhamnopyranosyl-*β*-D-glucopyranoside)	270 mg/g CMA	[34]
		Cyanidin 3-O-*β*-D-glucopyranoside	233 mg/g CMA	[34]
		Cyanidin 7-O-*β*-D-glucopyranoside	33 mg/g CMA	[34]
		Pelargonidin-3- glucoside	NA	[37]
		Pelargonidin-3-rutinoside	NA	[37]
		Petunidin 3-O-*β*-glucopyranoside	5.1 mg/g CEE	[38]
	Flavonols	Rutin	0.065–7.728 mg/100 g FW	[39]
		Myricetin	0.66–1.18 mg/100 g DW	[40]
		Quercetin	31.88–58.42 mg/100 g DW	[40]
		Quercetin 3-O-glucoside	1.069 mg/100 g FW	[29]
		Quercetin 3-O-rutinoside	2.869 mg/100 g FW	[29]
		Quercetin 3-O-galactoside	0.002 mg/100 g FW	[29]
		Kaempferol	0.24–1.61 mg/100 g DW	[40]
		Kaempferol 3-O-rutinoside	2.00–14.00 mg/100 g DW	[18]
		Kaempferol 3-O-glucoside	1.623 mg/100 g FW	[29]
	Flavanols	Catechin	309.26–750.01 mg/100 g DW	[40]
		Epicatechin	8.47–17.12 mg/100 g DW	[40]
		Epigallocatechin gallate	0.033–0.086 mg/100 g DW	[39]
		Procyanidin B1	59.64–224.41 mg/100 g DW	[40]
		Procyanidin B2	1.02–5.66 mg/100 g DW	[40]

MAE, mulberry anthocyanin extract; NA, not available; CEE, crude ethanol extract; CMA, crude mulberry anthocyanin; DW, dry weight; and FW, frozen weight.

The article "Assessing the Nutritional-Value-Based Therapeutic Potentials and Non-Destructive Approaches for Mulberry Fruit Assessment: An Overview" was retracted in 2023. Reasons: unreliable results or conclusions; concerns about the data; concerns about the peer review; concerns about the citations.

**Table 3:** Composition of phenolic acid in mulberry fruit.

Class	Subclass	Compound	Content	References
Phenolic acid	Hydroxycinnamic acid	Chlorogenic acid	5.3–17.3 mg/100 g DW	[48]
		Cinnamic acid	11.63–15.04 mg/100 g DW	[40]
		p-Coumaric acid	0.024–0.142 mg/100 g DW	[39]
		o-Coumaric acid	0.015 mg/g FW	[22]
		Ferulic acid	0.057–2.949 mg/100 g DW	[39]
		Caffeic acid	1.06–8.17 mg/100 g DW	[40]
	Benzoic acid	p-Hydroxybenzoic acid	0.028–0.154 mg/100 g DW	[39]
		Protocatechuic acid	0.264–0.794mg/100 g FW	[39]
		Gallic acid	7.34–23.35 mg/100 g DW	[40]
		Vanillic acid	0.008 mg/g FW	[22]
		Syringic acid	0.049 mg/g FW	[22]

FW, frozen weight and DW, dry weight.

**Table 4:** List of isolated polysaccharides from the mulberry fruit.

Compound name	Molecular weight	Bioactivities	References
FMAP	130	—	[53]
MP	—	Anti-apoptotic and anti-inflammatory	[54]
PMF-1	71.68	—	[55]
PMF-2	84.33	—	
PMF-3	103.17	—	
MFP	—	Hypoglycemic and anti-oxidant	[56]
MFP-1	—	Hypoglycemic and anti-oxidant	
MFP-2	—	Hypoglycemic and anti-oxidant	
MFP-1	7.9, 1.0, 0.7	Hypoglycemic and anti-oxidant	[35]
MFP-2	149, 9.3, 2.6.1.5	Hypoglycemic and anti-oxidant	
MFP-3	167, 5, 1.5	Hypoglycemic and anti-oxidant	
MFP-4	185, 64.4, 1.5, 0.2	Hypoglycemic and anti-oxidant	
MFP3P	136.6	Hypoglycemic and anti-oxidant	[57]
JS-MP-1	1639	Anti-obesity and immunomodulation	[58]

**Table 5:** Therapeutic properties of mulberry fruit.

Therapeutic properties	Intake type	Bioactive compounds	Health effects	References
Hypolipidemic	Mulberry freeze-dried powder	Fatty acids, dietary fiber, phenolics, anthocyanins, flavonoids, and vitamins	A significant decline in serum and liver triglyceride levels, total cholesterol, serum low-density lipoprotein cholesterol, and a decrease in the atherogenic index, while the serum high-density lipoprotein cholesterol was significantly increased	[70]
	Mulberry water extract	Phenolics, anthocyanins, flavonoids, and vitamins	Significant reduction in the levels of low-density lipoprotein, cholesterol, and triglyceride	[71]
	Mulberry freeze-dried powder	Anthocyanins	Significant reduction in the low-density lipoprotein cholesterol and total cholesterol	[72]
Anti-atherosclerotic	Mulberry water extract	Phenolics, anthocyanins, flavonoids, and vitamins	Significant decrease in severe atherosclerosis in the aorta by 42–63%	[71]
Anti-diabetic	Ethyl acetate-soluble extract	Phenolic compounds (25 different types)	Significant reduction in the glycosylated serum protein and fasting blood glucose and increase anti-oxidant enzymatic activities (SOD, CAT, GSH-Px) in streptozotocin (STZ) induced diabetic mice	[73]
	Mulberry fruit polysaccharides extract	Polysaccharides	Significant reduction in fasting blood glucose, oral glucose tolerance test, fasting serum insulin levels, homeostasis model of assessment-insulin resistance, glycated serum protein, and triglycerides	[74]
	Mulberry anthocyanin extract	Anthocyanin	Significant improvement in the dysfunction in diabetic mice and mitigated insulin resistance in HepG2 cells via activation of PI3K/AKT pathways	[75]
	Ramulus mori polysaccharides extract	Ramulus mori polysacchguoarides	Blood glucose-lowering and metabolism-normalizing roles and also improvement in the function of the pancreas by inhibiting the inflammatory response and attenuating the oxidative stress in pancreas tissue	[76]
Anti-obesity	Mulberry water extracts	Gallic acid, chlorogenic acid, rutin, and anthocyanins	Regulation of lipolysis and lipogenesis, which exerted the hypolipidemic and anti-obese effects	[77]
	Mulberry leaf extract and mulberry fruit extract	Cyanidin-3-glucoside, 1-deoxynojirimycin, rutin, and resveratrol	Potential anti-obesity effects through modulation of oxidative stress and obesity-induced inflammation in high fat diet-induced obesity	[78]
Anti-tumor	Mulberry anthocyanins rich extract	Anthocyanin	Targeting c-jun and p38/p53 pathways suppress tumorigenesis and cell survival but produce apoptotic death in AGS cells	[79]
Hepatoprotective	Extract	Anthocyanin	Potent protective effect on CCl4-induced liver fibrosis in rats	[80]
	Mulberry anthocyanin extract	Anthocyanin	Occurrence of the hypolipidemic effects of mulberry anthocyanin extract via inhibition of lipid biosynthesis, phosphorylation of AMPK, and stimulation of lipolysis	[81]
Neuroprotective	Mulberry extract	Cyanidin-3-O-beta-d-glucopyranoside	Neuroprotective effects on the PC12 cells exposed to hydrogen peroxide in vitro and on cerebral ischemic damage in vivo	[82]
Protective against cytotoxicity and oxidative stress	Mulberry juice purification and mulberry marc purification	Total flavonols, total phenolic acids, and anthocyanins contents	Potent anti-oxidant and anti-fatigue properties	[83]

The article "Assessing the Nutritional-Value-Based Therapeutic Potentials and Non-Destructive Approaches for Mulberry Fruit Assessment: An Overview" was retracted in 2023. Reasons: unreliable results or conclusions; concerns about the data; concerns about the peer review; concerns about the citations.

**Table 6:** Anti-oxidant potential of mulberry fruit measured through various methods.

Species	ORAC, mmol TE g^−1^	ABTS, mg TE 100g^−1^	FRAP, mg TE 100g^−1^	DPPH, mg TE 100g^−1^	Cuprac, mg TE 100g^−1^	References
Black mulberry	Nr	2,788.0	1,836.0	946.0	4,046.0	[31]
	Nr	0.68–1.44	0.73–1.69	Nr	Nr	[89]
	Nr	Nr	Nr	11.5–14.5	Nr	[90]
Red mulberry	Nr	0.51–0.73	0.37–0.77	Nr	Nr	[89]
	0.301–1.728	Nr	Nr	Nr	Nr	[91]
White mulberry	Nr	Nr	Nr	29.19–44.71	Nr	[92]
	Nr	Nr	Nr	10.7–12.9	Nr	[90]
Different cultivars	Nr	0.44–1.39	Nr	Nr	Nr	[22]
	Nr	0.0384–0.2073	Nr	0.0362–0.1291	Nr	[18]
Ten cultivars of red, black, and white mulberry	Nr	1.0–325.55	Nr	1.0–160.0	Nr	[29]

Nr: not reported.

## Data Availability

The data set supporting the conclusions of this article is included within the article.
